# Image Recognition and Encryption Algorithm Based on Artificial Neural Network and Multidimensional Chaotic Sequence

**DOI:** 10.1155/2022/9576184

**Published:** 2022-08-05

**Authors:** Shujun Fang, Xin Chen

**Affiliations:** ^1^ School of Computer Science and Engineering Northeastern University Shenyang 110819, China, neu.edu.cn; ^2^ School of Software and Microelectronics Peking University 24th Jinyuan Road Daxing Industrial District Beijing 102600, China, pku.edu.cn

## Abstract

With the continuous development of Internet technology and technological innovation, image recognition technologies such as face unlocking and face brushing payment have gradually entered daily life. However, it can not be ignored that these technologies not only bring us great convenience but also face great risks. The biological characteristics of a face image are unique, and it will be difficult to modify once it is leaked. If the image information stored in the cloud is leaked because it cannot be properly kept, users have no privacy. The encryption and recognition of face image can effectively solve this problem. Aiming at this, high‐dimensional chaos Henon Map and one‐dimensional chaos Logistic Map are used to generate a key to complete the encryption of the image in the transformation domain, and the capacity and complexity of the key are further enhanced. Then, combined with BP neural network to achieve face image recognition. Finally, the robustness of the proposed algorithm is verified and analyzed by conventional attacks, geometric attacks, and occlusion attacks.

## 1. Introduction

With the continuous development and progress of Internet technology, information security and privacy protection have attracted more and more attention [1–7]. The development of scientific and technological revolution has promoted the advent of the Internet era, and computer intelligent image recognition technology is becoming more and more mature [8–11]. Face recognition, which is an important field in image recognition, is a biometric technology for identity recognition based on facial features [5, 12, 13]. It is a research hotspot of artificial intelligence and computer vision. It is widely used in the fields of access control system, financial payment, public security, and so on. The process of traditional authentication methods such as ID card, password, and signature is cumbersome. When users forget to carry relevant certificates or forget the password, it will bring a series of unnecessary troubles, and these methods are easy to be tampered with and forged. Compared with other biometric recognition methods such as iris recognition and fingerprint recognition, the advantage of face recognition is noncontact and nonmandatory. Users do not need to contact the device directly. The recognized face image information is actively obtained by the device, and the recognition process is more friendly. At present, most of the research on face recognition is based on the plaintext domain, and there is little research on encrypted face recognition. In order to effectively protect face image data, it is of great significance to study encrypted face image recognition.

Discrete wavelet transform (DWT) [14, 15] has better spatial‐frequency domain decomposition characteristics than other frequency‐domain transforms, but its antiattack ability is poor. For this reason, we study an encrypted face recognition algorithm based on a neural network [16] and DWT‐Discrete Cosine Transform (DWT‐DCT) transform [17] and propose an image recognition and encryption algorithm based on an artificial neural network and multidimensional chaotic sequence.

## 2. Encryption Method

The encryption process of the encrypted face image recognition algorithm based on neural network and DWT‐DCT transformation is shown in Figure 1.

**Figure 1:** The encryption process of the encrypted face image recognition algorithm.

The detailed encryption steps are as follows:

(1) Use wavelet transform to decompose the face image *f*(*i*, *j*) with a two‐layer wavelet, and obtain 4 sub‐band matrices [LL, HL, LH, HH];
(1) LL,HL,LH,HH=DW  T2fi,j.
(2) Perform DCT transformation on the four sub‐band matrices, respectively, to obtain sub‐band frequency domain coefficient matrices: LL1, HL1, LH1, and HH1;
(2) LL12=DCTLL,HL12=DCTHL,LH12=DCTLH,HH12=DCTHH.
(3) The chaotic sequence is generated by the Henon map and Logistic map, respectively, and the chaotic sequence is binarized to obtain the binarized matrix *H*(*i*, *j*) and *L*(*i*, *j*);
(4) XOR the binary matrix to obtain the encrypted binary matrix *S* ^′^(*i*, *j*);
(3) S′i,j=Hi,j⊗Li,j.
(5) Set the 0 element in S^′^(i, j) to ‐1, and construct the encrypted binary matrix S(i, j) according to the size of the image;
(6) Do point multiplication with the encrypted binary matrix S(i, j) and the sub‐band frequency domain coefficient matrix LL1, HL1, LH1, and HH1 to complete the face image encryption in the frequency domain;
(4) ELL=Si,j⋅∗LL1,EHL=Si,j⋅∗HL1,ELH=Si,j⋅∗LH1,EHH=Si,j⋅∗HH1.
(7) Then, carry out IDCT transformation on ELL, EHL, ELH, and EHH to get the encrypted sub‐band matrix ELL1, EHL1, ELH1, and EHH1;
(5) ELL12=I  DC  TELL,EHL12=I  DC  TEHL,ELH12=I  DC  TELH,EHH12=I  DC  TEHH.
(8) Finally, perform IDWT transformation on the encrypted sub‐band matrix to obtain the encrypted face image E(i, j);
(6) Ei,j=I  DW  T2ELL1111,EHL,ELH,EHH,

### 2.1. Encryption Effect

The images before and after encryption by Logistic Map [18–20] and Henon Map [21–23] are shown in Figure 2. It can be seen from the image effects before and after encryption that the encrypted image has a good encryption effect, which can effectively protect image data under the condition that the key is not leaked.

**Figure 2:** The Original Images and corresponding encrypted images.

### 2.2. Sensitivity Analysis

During the experiment, the parameter values of Henon mapping are selected as follows, *a* = *l*.5, *b* = 0.323, *X*_0_  = 0.76235607, *Y*_0_ = 0.2236674091, the growth parameter of Logistic mapping is 4, and the initial value *X*_0_ = 0.122. Taking the first expressive face of the first person in the ORL face database as the test object to test the sensitivity. Due to the limited computational precision of the computer, there will be some data loss in the encryption and decryption of the frequency domain transform, and the image decrypted by the correct key will be slightly different from the original image, but overall the same.

It can be seen from the decrypted images that even if a slight change in the key cannot decrypt the image correctly, causing the decryption to fail, indicating that the encryption method is highly sensitive.

### 2.3. Correlation Analysis

Correlation analysis is also a kind of data analysis attacks. Generally, the correlation between adjacent pixel values of any plaintext image is strong, whether in the horizontal direction, vertical direction, or diagonal direction. If the encryption effect is good, the correlation between adjacent pixel values in these three directions is relatively weak. The calculation formula of the correlation coefficient between adjacent pixels is

(7) C=∑n=1Nxn−x¯yn−y¯∑n=1Nxn−x¯2∑n=1Nyn−y¯2,

where *N* represents the logarithm of randomly selected adjacent pixels, *x*(*n*) and *y*(*n*) are pixel values of randomly selected adjacent pixel pairs.

(8) x¯=1N∑n=1Nxny¯=1N∑n=1Nn

In order to more clearly see the difference between encrypted image and plaintext image, plaintext image Einstein will be used as a test image to test the correlation coefficient of encrypted image and plaintext image in three directions. Figure 3, respectively, shows the correlation distribution Figure 4 of plaintext image and Figure 5ciphertext image in horizontal, vertical, and diagonal directions.

Figure 3The correlation distribution of plaintext image (a) and ciphertext image (b) in a horizontal direction.

**Figure:** (a)

**Figure:** (b)

Figure 4The correlation distribution of plaintext image (a) and ciphertext image (b) in a vertical direction.

**Figure:** (a)

**Figure:** (b)

Figure 5The correlation distribution of plaintext image (a) and ciphertext image (b) in a diagonal direction.

**Figure:** (a)

**Figure:** (b)

Through the test of multiple images, the test values of the correlation coefficient between the plaintext image and the corresponding ciphertext image in three directions show that the value of the correlation coefficient of the ciphertext image in three directions is close to 1, while the value of the correlation coefficient of the ciphertext image in the corresponding direction is close to 0, and some even show a negative correlation. Therefore, the plaintext image eliminates the correlation between adjacent pixel values under the action of the encryption algorithm, so that the attacker cannot obtain directly valuable information.

## 3. Algorithm Flow

The specific flow of the proposed image recognition and encryption algorithm based on an artificial neural network and multidimensional chaotic sequence is shown in Figure 6.

**Figure 6:** The specific flow of the proposed image recognition and encryption algorithm.

The detailed identification steps are as follows:

(1) Encrypt the image in the DWT‐DCT transform domain for the original image database
(2) Using the PCA algorithm to extract the characteristics of the encrypted image of the training sample and obtain the projection matrix *T*
(3) The dimension reduction matrix *D* is obtained by projecting the training sample *X* through the projection matrix *T*
(4) Use the dimensionality reduction matrix *D* as the input of the neural network to create and train the neural network
(5) Use the proposed encryption method to encrypt the face to be tested to obtain the encrypted image *E*_1_
(6) Project the encrypted image *E*_1_ through the projection matrix *T* to obtain the dimension‐reduced face matrix *E*_2_
(7) Input the dimensionality reduction face matrix *E*_2_ into the trained neural network to complete the recognition of the face to be tested

## 4. Experiment

### 4.1. Recognition Rate

In constructing the BP neural network [24–26], the input of the BP neural network is also different with different energy selected, and the recognition rate of the encryption algorithm will be different. During the experiment, the influence of the energy coefficient on the recognition rate of the neural network was analyzed by changing the size of the energy coefficient. The recognition rates of encrypted face recognition algorithms based on neural network and DWT‐DCT transform under different energy coefficient conditions are shown in Table 1. Table 1 shows that when the selected energy coefficient is 75, the recognition rate of the encryption algorithm at this time is 63.5%. When the energy coefficient chosen increases gradually, the recognition rate of the encryption algorithm will also increase accordingly. When the energy coefficient goes 85%, the eigenvectors corresponding to the first 48 largest eigenvalues are selected, the projection matrix is 10315∗48, the input after dimension reduction is 200∗48, and the recognition rate of the encryption algorithm goes to the maximum value of 82%. Then, as the energy coefficient increases, the recognition rate of the encryption algorithm will decrease correspondingly. It can be seen that the more significant the selected energy coefficient, the better, and the more retained eigenvectors, the better. Only by selecting appropriate energy coefficients and eigenvectors can the performance of the encryption algorithm be optimal.

**Table 1:** Image recognition rate of encryption algorithm under different energy coefficients.

Energy coefficients (%)	75	80	85	90	95
Eigenvectors (number)	24	32	48	71	114
Recognition rate (%)	63.5	74.5	82	80.5	78.7

In the simulation experiment, the face image of the first person in the ORL face database is selected as the test image to test the robustness of the encrypted face recognition algorithm based on neural network and DWT‐DCT transformation. Before the experiment, 50 people in the ORL face database were marked as serial numbers 1–50. The face images to be tested were subjected to conventional attacks, geometric attacks, lighting attacks, occlusion attacks, and others. The robustness of the encryption algorithm is evaluated by testing whether the image to be tested can still be accurately recognized after being attacked.

### 4.2. Conventional Attack

#### 4.2.1. Gaussian Noise

During the experiment, the function imnoise() of Matlab is used to add Gaussian noise to the image to be tested. The data obtained from the experiment are shown in Table 2.

**Table 2:** The experiment data after Gaussian noise attack.

Noise intensity (%)	5	10	15	20	25
PSNR (dB)	12.86	10.11	9.24	8.77	8.21
Identification number	1	1	1	1	1

Observing the data in Table 2, it can be concluded that when the Gaussian noise attack intensity increases from 5% to 25%, the PSNR value of the image drops from 12.86 to 8.21. At this time, the image is quite blurred and difficult to see visually.

However, the proposed encryption algorithm can always accurately identify the person whose serial number is 1, indicating that this chapter′s encryption algorithm has good antiattack ability against Gaussian noise attacks.

#### 4.2.2. JPEG Compression

A JPEG compression experiment was performed on the face image to be tested, and the compression quality was used to describe the degree of image compression. The smaller the compression quality, the higher the compression degree of the image, and the worse the image quality. The purpose of image compression is achieved by selectively removing high‐frequency redundant parts.

The data obtained in the experiment after the JPEG compression attack are shown in Table 3.

**Table 3:** The experiment data after JPEG compression attack.

Compression quality (%)	5	10	15	20	25
PSNR (dB)	22.34	25.56	27.88	29.42	29.75
Identification number	1	1	1	1	1

Observing at Table 3, it can be seen that when the compression quality is 5, the PSNR value of the image is 22.34, the image has become quite blurred and difficult to identify, but the encryption algorithm can still accurately identify the face image with serial number 1. When the compression quality increases gradually, the PSNR value of the image will increase progressively, and the degree of distortion will become lower and lower. When the compression quality is 25, the PSNR value at this time is 29.75. The proposed encryption algorithm recognizes the encrypted face image as the person whose serial number is 1 in the ORL face database. To sum up, the proposed image recognition and encryption algorithm based on an artificial neural network and multidimensional chaotic sequence has good resistance to JPEG attacks.

#### 4.2.3. Median Filter

Median filtering is a nonlinear processing technology that reorders the gray values in the field according to their size. It selects the median value of the ordered sequence as the output pixel value, which can overcome the blurring of image details caused by linear average filtering. The filter window size is [7 × 7], and the face image with 10 times of filtering is tested, and the specific experimental data obtained in the experiment are shown in Table 4.

**Table 4:** The experiment data with median filter.

Parameter	[3 × 3]			[5 × 5]			[7 × 7]		
Frequency	1	5	10	1	5	10	1	5	10
PSNR (dB)	31.44	29.71	29.03	28.66	24.32	24.01	26.55	22.34	20.76
Identification number	1	1	1	1	1	1	1	1	1

Observing Table 4, it can be seen that as the number of filters or the filter window increases, the PSNR value of the image will decrease, and the proposed encryption algorithm can always accurately identify the face image with serial number 1. The encryption algorithm has an excellent antiattack ability to median filter.

### 4.3. Geometric Attack

#### 4.3.1. Translation Attack

Under the condition of translation attack, the image is moved up and down, left and right, and the antitranslation attack ability of the encryption algorithm is tested by changing the percentage coefficient of translation. The experimental data obtained by horizontal left shift and horizontal right shift are shown in Table 5.

**Table 5:** The experiment data with horizontal attack.

	Horizontal left				Horizontal right			
Move percentage (%)	30	31	32	33	8	9	10	11
PSNR (dB)	8.57	8.34	8.25	8.13	14.44	13.36	13.11	12.52
Identification number	1	1	20	20	1	1	15	15

Observing Table 5, it can be seen that before the horizontal left shift percentage goes 32%, the encryption algorithm can accurately identify the face with serial number 1. When the left shift percentage is 32%, it has suffered a considerable strength attack. The PSNR value of the image is 8.25, the encryption algorithm cannot accurately recognize the face, and it will be mistakenly identified as the person whose serial number is 20. The horizontal right shift can be accurately recognized until the horizontal right shift percentage goes 10%. When the right shift percentage goes 10%, the PSNR is 13.11 at this time, and the encryption algorithm will incorrectly identify the face image for the person whose serial number is 15 in the ORL face database. It is not difficult to see that the ability of the proposed algorithm to resist a horizontal left shift attack is obviously better than that of a horizontal right shift attack.

The experimental data obtained by moving the face image to be tested vertically up and down are shown in Table 6.

**Table 6:** The experiment data with vertical attack.

	Vertical up				Vertical down			
Move percentage (%)	5	6	7	8	4	5	6	7
PSNR (dB)	14.78	14.06	13.45	13.11	18.57	17.78	16.35	16.02
Identification number	1	1	19	19	1	1	17	17

Observing the data in Table 6, it can be seen that the encryption algorithm has almost the same resistance to vertical upward and vertical downward attacks. When the vertical upward movement percentage is less than 7%, it can accurately identify the person with serial number 1. When the moving percentage reaches 7%, the encryption algorithm will incorrectly identify the person with serial number 19. When the percentage of vertical downward movement goes 6%, the PSNR value of the image will be 16.35, and it will be mistakenly identified as the person with the serial number 17. It can be seen that the encrypted face recognition algorithm has the same resistance to vertical up and vertical down.

#### 4.3.2. Rotation Transformation

In the experiment, the rotation angle change is used as the change parameter, and the face image to be tested is rotated clockwise and anticlockwise to test the antirotation attack ability of the proposed encrypted face image recognition algorithm.

The experimental data obtained after clockwise rotation and anticlockwise rotation are shown in Table 7.

**Table 7:** The experiment data with rotation attack.

	Clockwise rotation				Anticlockwise rotation			
Degree of rotation (°)	11	12	13	14	12	13	14	15
PSNR (dB)	15.48	15.17	14.89	14.63	15.16	14.87	14.62	14.89
Identification number	1	1	5	5	1	1	2	2

It can be seen from Table 7 that the PSNR value of the image is inversely proportional to the degree of rotation. When the degree of clockwise or anticlockwise rotation increases, the PSNR value of the image will decrease accordingly. When the clockwise rotation goes 13°, the encryption algorithm can be accurately identified. When the rotation degree increases to 13°, the PSNR value is 14.89. The person with serial number 5 will be wrongly identified at this time. For anticlockwise rotation, when the degree of rotation increases to 14°, the encrypted face recognition algorithm will incorrectly identify the person with the serial number 2. It can accurately identify the person with the serial number 1 before that. The proposed encrypted face recognition algorithm has the same resistance to clockwise rotation as anticlockwise rotation.

### 4.4. Light Attack

During the experiment, Photoshop software was used to simulate the lighting conditions to preprocess the image. The antilight attack ability of the encrypted face recognition algorithm was tested by changing the light intensity. The experimental data under different illumination conditions are shown in Table 8.

**Table 8:** The experiment data with light intensity.

Light intensity (%)	−90	−60	−30	30	60	90
PSNR (dB)	11.35	14.87	22.13	23.41	15.67	11.81
Identification number	1	1	1	1	1	1

Observing the data in Table 8, it can be seen that when the intensity of the light attack changes from strong to weak and then strong, the PSNR value of the image will decrease as it increases. In this change process, the encrypted face recognition algorithms proposed in this chapter can be accurately identified as the person whose serial number is 1, which indicates that the encrypted face recognition algorithm based on the network and DWT‐DCT transformation has good resistance to light attacks.

### 4.5. Occlusion Attack

In real life, face images will inevitably be occluded by masks, glasses, hats, etc., and occlusion will significantly impact face recognition. In the experiment, Photoshop software is used to preprocess the image to be tested and simulate the occlusion of masks, glasses, and hats to test the resistance of the encrypted face recognition algorithm to occlusion attack.

The experimental data after being occluded by different occlusion areas are shown in Table 9.

**Table 9:** The experiment data with different occlusion.

Occlusion	Occluded by glasses			Occluded by mask			Occluded by hat		
	Small	Middle	Large	Small	Middle	Large	Small	Middle	Large
PSNR (dB)	18.89	17.22	15.43	18.78	17.21	15.41	12.78	11.66	10.81
Identification number	1	1	21	1	1	1	25	25	25

From the data in Table 9, it can be seen that for the occlusion of glasses, the person with the serial number 1 can be accurately identified before the occlusion area reaches Large. When the occlusion area is further expanded to *L*, it will be incorrectly recognized as the person with serial number 21 in the ORL face database. For mask occlusion, the encrypted face recognition algorithm can always accurately recognize, while the hat occlusion is always incorrectly recognized as the person with serial number 25. This shows that the designed algorithm has good resistance to glasses occlusion and mask occlusion, while the resistance to hat occlusion is relatively poor.

## 5. Analysis and Discussion

The recognition rates of three algorithms (unencrypted, DCT, DFT, and DWT‐DCT) are compared with the recognition rates of the algorithms without encryption. The face image recognition rates of various algorithms under different energy coefficients are shown in Figure 7.

**Figure 7:** The image recognition rates of various algorithms under different energy coefficients.

It can be seen from the data in Figure 7 that the recognition rates of the three encrypted face image recognition methods are different under different energy coefficients.

When the selected energy coefficient reaches 85%, the recognition rate of the encrypted face recognition algorithm based on DCT transform and DWT‐DCT transform reaches the maximum, which are 80% and 81%, respectively, and the difference between the recognition rate of the algorithm without encryption and 82% is only within 2%. The maximum recognition rate of the encrypted face image recognition algorithm based on the DFT transform appears at the energy coefficient of 95%, reaching 81%.

For different encrypted face recognition algorithms, it is necessary to select the appropriate energy coefficient to optimize the algorithm’s performance. The security of face image data is effectively protected after chaotic encryption.

## 6. Conclusions

This paper proposes an image recognition and encryption algorithm based on an artificial neural network and multidimensional chaotic sequence. It adopts the combination of high‐dimensional chaos and one‐dimensional chaos to enhance the security of the key. And, complete the image encryption in the DWT‐DCT transform domain and use PCA and BP neural network to achieve face recognition. Then, the key sensitivity, algorithm recognition rate, and robustness of the encryption algorithm were analyzed and tested. Finally, the algorithm recognition rate and robustness of the three encrypted face recognition algorithms and unencrypted face recognition are compared and analyzed. The results show that the recognition rate of the face recognition method using transform domain encryption is not much different from that of the unencrypted face recognition method, and it has good robustness. And, after encryption, the security of face image data on the Internet is greatly improved.

## Conflicts of Interest

The authors declare that they have no conflicts of interest.

## Data Availability

The data used to support the study are included in the paper.
